RETRACTED

# A Novel Text Mining Approach for Mental Health Prediction Using Bi-LSTM and BERT Model

**DOI:** 10.1155/2022/7893775

**Published:** 2022-03-03

**Authors:** Kamil Zeberga, Muhammad Attique, Babar Shah, Farman Ali, Yalew Zelalem Jembre, Tae-Sun Chung

**Affiliations:** ^1^Department of Artificial Intelligence, Ajou University, Suwon, Republic of Korea; ^2^Department of Software, Sejong University, Republic of Korea; ^3^College of Technological Innovation, Zayed University, Abu Dhabi, UAE; ^4^Department of Electronic Engineering, Keimyung University, Daegu, Republic of Korea

## Abstract

With the current advancement in the Internet, there has been a growing demand for building intelligent and smart systems that can efficiently address the detection of health-related problems on social media, such as the detection of depression and anxiety. These types of systems, which are mainly dependent on machine learning techniques, must be able to deal with obtaining the semantic and syntactic meaning of texts posted by users on social media. The data generated by users on social media contains unstructured and unpredictable content. Several systems based on machine learning and social media platforms have recently been introduced to identify health-related problems. However, the text representation and deep learning techniques employed provide only limited information and knowledge about the different texts posted by users. This is owing to a lack of long-term dependencies between each word in the entire text and a lack of proper exploitation of recent deep learning schemes. In this paper, we propose a novel framework to efficiently and effectively identify depression and anxiety-related posts while maintaining the contextual and semantic meaning of the words used in the whole corpus when applying bidirectional encoder representations from transformers (BERT). In addition, we propose a knowledge distillation technique, which is a recent technique for transferring knowledge from a large pretrained model (BERT) to a smaller model to boost performance and accuracy. We also devised our own data collection framework from Reddit and Twitter, which are the most common social media sites. Finally, we employed word2vec and BERT with Bi-LSTM to effectively analyze and detect depression and anxiety signs from social media posts. Our system surpasses other state-of-the-art methods and achieves an accuracy of 98% using the knowledge distillation technique.

## 1. Introduction

The automatic detection of mental health conditions is one of the most important and complex health concerns in the real world. Mental health affects the behavior, thinking, and mood of individuals interacting with the world around them. In addition, mental health problems are becoming a leading disability, contributing largely to the universal burden of disease. In general, the number of people with signs of depression in 2015 was projected to be 4.4% (more than 332 million people) [1]. As reported in a WHO study, depression is a shared universal mental disorder that affects a large number of people regardless of their age. There are many limitations in depression recognition and treatment, including a lack of professionals in the health sector, social shaming, or an inappropriate diagnosis. Prolonged depression and anxiety can lead to suicide if the affected individual is not provided good care and immediate help. In addition, depressive disorders have been categorized as one of the largest contributors to nonfatal health loss. Suicide has become a major reason for death among young people with a general suicide rate of 10.5 per 100,000 people, which is nearly 800,000 cases every year in absolute measure [2, 3].

RETRACTED

The rapid integration of smart sensors in hand phones and wearable devices has increased access to intelligent mental healthcare, permitting the gathering of measurable signs in a clear and modest way, giving a reasonable estimate of the physical and psychological states of users [4, 5]. Many types of sensors can be incorporated into the mental healthcare process and can provide accurate, momentary, and continuous patient data [6]. Until recent days, many systems in the medical sector were designed to supervise the mental health of users using smartphones and wearable sensors as a data source [4, 7]. However, such systems are not positioned to gather valuable information on demand keeping the freshness of data. It is also known that digital devices yield a large portion of mental-health-problem-related data, which are not enough to efficiently supervise patients. Moreover, obtaining meaningful information from these data and efficiently examining them has become extremely challenging for traditional mental health problem detection systems.

Social media has recently become a persuasive tool to inspect the mental health and mental state of the users, particularly the youth. It also provides anonymous contributions in numerous online platforms to leave room for open dialog regarding socially defamed topics and motivate users to fight against mental health problems [8]. In addition, patients can share their ideas about the recent common health problems. Healthcare monitoring systems for the detection of depression and anxiety can apply social media data to recognize the mental state of users based on their posts and comments. However, the data published on social networking sites on mental-health-related problems contain unstructured, unpredictable data composed of idioms, jargon, and dynamic topics. Thus, it is becoming very difficult for an application to fetch the desired data about patients and evaluate them to confirm that they receive the proper treatment they need as early as possible. As a result, there should be a smart approach that is capable of retrieving the most valuable data features with a minimal dimensionality that maximizes the accuracy of systems in the healthcare environment on mental health.

RETRACTED

Machine learning algorithms such as decision trees, support vector machines (SVMs), logistic regression, AdaBoost, and multilayer perceptron (MLP) have been used to support doctors in diagnosing symptoms of depression and anxiety [9–13]. However, unremitting patient monitoring gives a large portion of health-related data containing voice patterns, textual data, sensor data, and emojis, all of which have increased significantly [14]. The existing systems that apply machine learning are not capable of dealing with these types of data to precisely get meaningful evidence and cannot capture semantic significance in text posts disseminated in social media. Moreover, such data will remain useless for healthcare businesses until they are managed and classified wisely in time-sensitive manner [15, 16]. This demands a smart approach that can accurately classify the textual data related to mental health problems [3, 9, 17, 18].

The concept of deep learning addressed many key issues in natural language processing tasks such as sentiment analysis, and the current sentiment analysis on social media content is increasingly focused on the use of new deep learning architectures and models for mental problem identification and classification [19–21]. However, the new development in health sector systems poses a huge burden for researchers because they require collaboration with interdisciplinary steps, new technologies, and changes in society. As a result, these previous healthcare systems are inefficient and ineffective in coping with these new trends.

This study proposes a smart and context-aware deep learning framework based on bidirectional encoder representations from transformers (BERT) to effectively identify mental-health-related problems from user posts on social media with improved classification accuracy. This study combines different sources of information for an efficient analysis of mental-problem-related data. We have adopted a knowledge distillation scheme to transfer knowledge from large pretrained BERT to a smaller model and used bidirectional long short-term memory (Bi-LSTM) to examine depression- and anxiety-related data. The results indicate that our presented system precisely handles the mixed data and enhances the performance of mental health classification. In general, our key contributions to this research work are fourfold:

- A new framework is presented to extract a huge size of highly appropriate depression- and anxiety-related data from Twitter and Reddit. In addition, we implemented a combined cyber-community-group-based labeling and keyword-based data crawling technique based on the circumplex model of emotion to identify the desired mental health problem data.
- A deep neural network-based bidirectional text representation model, that is, BERT, is used to embody mental health problem textual data maintaining contextual and semantic connotations. In addition, we proposed a sequence processing model called bidirectional long short-term memory (Bi-LSTM) as a classifier, which effectively maximizes the amount of information accessible to the network, improving the content available to the algorithm in knowing what words immediately follow and come before a given word in a sentence.
- We propose a knowledge distillation technique, which is a means of transferring knowledge from a large pretrained model (BERT) to a smaller model to maximize performance and accuracy. We filtered the large network (BERT) into another much smaller network (Distiled_BERT) for mental health-related problem identification, and it performs very well by transferring the required domain knowledge and applying it to a specific healthcare environment.
- We conducted extensive experiments using a principal component analysis (PCA) and different deep learning/ML models, the results of which are compared with other related models. This evaluation plays a key role in regulating the shortcomings of the already applied methods and classification models. The experimental results show that our model performs considerably well over the compared methods, which, after many hyperparameter optimizations, provides an accuracy of 98%.

RETRACTED

The remaining sections are organized as follows: Section 2 contains a description of mental health monitoring system using wearable devices and a deep learning approach.  Section 3 presents the whole framework proposed in this research.  Section 4 explains the results obtained in our experiment. Finally, in Section 5, we provide a conclusion of our study.

## 2. Related Studies

Machine learning (ML) models and big data play important roles in building a smart healthcare monitoring system for patients. Recently intelligent devices such as cellphones and many wearable sensors have been converged to generate the maximum evidence-based mental health data possible. Furthermore, the rapid growth of social media platforms and their application has increased at an unprecedented pace. This section discusses the detection of common mental illnesses based on wearable sensors using ML practices, social media data, and deep learning approaches using large sets of data.

### 2.1. Analysis of Mental-Health-Related Problems Using Wearable Sensors

The growing capacity of intelligent devices like cell phones makes them a prospective way for ecological momentary assessment measurements and the monitoring, treatment, and interventions of mental illness. This will reduce costs and help expand the mental health service for the larger societal group. The most commonly used smart devices in our day-to-day life such as cell phones and fitness bands contain sensors [22]. This extends the chance of many applications that consume information generated from sensors in the healthcare domain [23]. We can merge the data generated by these sensors to produce contextual information about patients regarding their mental status and social relationships [24]. Moreover, these types of multiple sensor integration have been used to get better results in different application areas compared to single sensors [25].

However, accumulated wearable sensor-based information exists in large volumes and is not well-structured. The previous research works did not apply innovative data processing techniques to get the desired latent information in them. Different studies, particularly on sensors, have been conducted on existing techniques to collect data, applying ML techniques to process the collected data [22]. Nevertheless, the previously proposed research works were not very successful in many different scenarios. Furthermore, mental health diagnosis is difficult to realize on a large scale because of the old data collection techniques such as interviews and questionnaires [26]. These approaches are unscalable to reach larger societal groups within a certain community. In addition, it is difficult to use them for knowledge extraction without designing an efficient and scalable system that can operate on a large set of data. Therefore, health organizations have moved away from conventional connections and now allow online group meetings for sharing information and seeking advice, thereby helping scale their approach to a certain extent. Recent studies have indicated that many social groups are willing to contribute and share ideas about health-related issues [9].

### 2.2. Analysis of Mental-Health-Related Problems Using Social Media Data with Machine Learning

Social media platforms recently are considered as backbones for the detection of mental health conditions. However, detecting depression through online social media is extremely challenging because it demands a well-designed and robust system that can deal with the complex nature of the data. It is very difficult to get an important and appropriate quantity of data related to mental illness. In recent years, the practice of utilizing social media data has boomed, and people started revealing their concerns without hesitation. This actually motivates researchers to conduct more research on the detection of health-related problems such as depression and anxiety as early as possible. In addition, data found in social media is replete with vague information, which mainly includes related metadata such as location, age, and other factors [27]. Kowsari et al. [28] proposed a deep learning model to analyze the mental status of patients based on Reddit posts. Many of the previous systems have applied insufficient data sets for depression and anxiety, which may produce imprecise results and thus perhaps mislead healthcare workers [29]. Artificial intelligence (AI) based techniques have been proposed to examine patients' posts on social media platforms and recognize serious problems in those patients [27]. An anxiety-related dictionary is constructed, and a given text is evaluated on the basis of the dictionary whether related to anxiety or not. However, the nature of texts posted on these platforms is always unorganized, and it is impractical to efficiently process them without using deep learning algorithms.

RETRACTED

Tadesse et al. developed the idea of processing a given post to check as to whether it contains the idea of suicide through deep learning and ML-based classification methods targeting Reddit data. The authors make use of an LSTM-CNN merged to compare it to different working approaches. There are commonly two steps to analyze social media data. First, data are collected from different sources such as networking sites, and the second task is to process the available data using statistical models. We proposed a combined cyber community-group-based labeling and keyword-based data crawling technique based on the circumplex model of emotion to identify the desired mental health problem data, as depicted in Figure 1 [30].

### 2.3. Deep-Learning-Based Text Embedding and Classification

Text representation is one of the underlying difficulties in sentiment analysis. The purpose of a text representation is to numerically denote unstructured text documents to make them mathematically commutable by maintaining the semantic and circumstantial meaning of the words in the text. Different ways of representing a given text corpus in a real-valued vector were studied and proposed by researchers [31]. Any given word in a text should be converted into a single vector so that it will be fed to the artificial neural network. As we can see from Figure 2, many studies have been conducted on word embedding techniques based on statistical methods for learning an individual word embedding from a text corpus such as word2vec, fastText, and GloVe. In addition, recent transformer-based deep learning techniques for representing words such as BERT, GPT, and GPT2 are extremely common [32, 33]. These models bring a major change to NLP downstream tasks by practicing predicting missing words in the text, and because they analyze every sentence with no specific direction, they do a better job at understanding the meaning of homonyms than previous ML approaches such as word embedding methods. Deep learning methods contain concurrent processing layers to represent data hierarchically and have exhibited good results in many domains. Young et al. reviewed many deep-learning-based practices that are used for various natural language processing (NLP) tasks [34]. Many recent studies have used deep learning to solve problems related to understanding the sole meaning of a given post, such as sentiment. However, all of these deep learning-based text representation techniques lack adequately labeled data sets for mental health problems. In addition, applying the best-fit word embedding approach to vectorize a very large data set has not been adequately addressed. We proposed a BERT-based text representation technique that efficiently and effectively captures the semantic meaning of words in a given text based on the attention mechanism [35].

RETRACTED

The other key challenge in dealing with sentiment analysis is the implementation of appropriate deep-learning-based classifier models. Researchers have implemented different classifier models, such as CNN and XGBoost, along with their own text-prepossessing techniques. The major challenge in NLP, in general, is capturing the semantic and syntactic meanings of a word in a largely given text corpus, which is generally termed as maintaining long-range dependency. Many studies have used a classical feature analysis, such as a CNN, an LSTM, and an LSTM-CNN merged to detect the idea of suicide in online forums [36, 37]. In this regard, the authors did not incorporate many recent deep learning techniques that deal with the representation of words along with their context. Researchers have also proposed a GRU and an LSTM-RNN, which are suitable for processing long textual data and applying them to the task of sentiment analysis [18, 38, 39]. Another interesting approach proposed by Burdisso et al. is a new way of dealing with texts, called smoothness, significance, and sanction (SS3), aiming to offer assistance for sentiment analysis in an integrated, easy, and efficient way. The classification process in most previous techniques was not self-explaining, and human beings are unable to naturally understand the motivations behind the classification [40]. The authors developed SS3 to address the incremental classification of chronological data and help with early classification and explainability. Nonetheless, most such research methods follow the same pattern when training the model. They first train their model on emotions using extracted textual data and then predict whether a given unobserved text is related to depression. Because the semantic and contextual relationships (long-term dependency) between words are properly captured, the models provide insufficient information and an inaccurate prediction. Therefore, their system attains minimal accuracy for sentiment classification.

RETRACTED

More recently, a range of model compression techniques has been established. We are using any model with the primary objective of making a very good generalization on unseen data after training it with a meaningful and sufficient data set. We need deeper models to train a large data set. However, we only need a lighter model that works well on any unobserved data set during testing. As a result, researchers have proposed knowledge distillation that effectively incorporates a smaller and light model from a large and complex model [34, 41]. As far as our research work is concerned, many research studies were done on mental health problems based on user posts. These studies do not leverage deep learning techniques and knowledge distillation effectively for representing collected texts [42, 43].

Finally, the attention mechanism has been one of the most significant developments in deep learning research during the last decade [44]. It has initiated the growth of many recent discoveries in NLP, including the transformer architecture [45] and Google's BERT [19]. Another comparable study associated with depression detection was conducted using a classification of news headlines, which used a manually annotated corpus [38, 45]. Xu et al. also presented long short-term memory (LSTM) neural network to obtain an appropriate meaning from large text [46]. From this literature, we see that researchers integrate classifiers differently with text embedding techniques and data sources to achieve a better result. However, we still need a more robust technique to automatically obtain sensible information from large text data posted on social media platforms keeping better accuracy.

RETRACTED

This work differs from existing studies in several aspects. First, many of the research works studied were not able to exploit the capability of context-aware deep learning framework based on bidirectional encoder representations from transformers (BERT) to effectively identify mental health-related problems from user's sentiment. Second, the application of knowledge distillation on top of deep learning enhances the effectiveness of our proposed model compared with many of the research works in this specific domain. Third, we have used multiple combinations of vectorization techniques that are listed in Figure 2 to make sure that our proposed approach performs better in maintaining long-term dependencies among a bag of words in a long text corpus that are posts from Reddit and Twitter in our case.

## 3. Proposed Framework

In this section, we present the framework intended to retrieve, process, evaluate, and classify social networking data about mental health such as depression and anxiety.  Figure 3 illustrates a general architecture that is proposed in this research work. Monitoring comments and posts on social media platforms can provide insights into how individuals self-reveal and talk about mental health issues. This type of information disseminated and shared across such platforms can be utilized as a data source for mental health problem identification. However, these types of data collected from social media are usually unstructured and include informal expressions, vague, and contentiously changing topics. It is extremely difficult to generate meaningful information from social media platforms that could be consumed in the domain of mental health evaluation and depression detection. Therefore, the proposed practical framework contains various modules such as data collection, data preprocessing, labeling techniques, word embedding, and classification. The primary objective of this research is to develop an automated system capable of discovering and evaluating mental health conditions using deep learning techniques such as BERT and Bi-LSTM. First, realtime data are extracted based on keyword-based queries from Twitter and Reddit using APIs (Tweedy and PRAW, respectively), as shown in Figure 3. After the desired number of data are gathered, different NLP techniques are applied to analyze the data (as depicted in task 2 of Figure 3. In addition, we examine the users' thoughts regarding depression and anxiety to categorize their mental health conditions as depression-related (positive) or standard posts (negative), as shown in task 3 in Figure 3. Text representation models, fastText, word2vec, and BERT, are used to embody the data with an appropriate vector. Finally, Bi-LSTM with softmax is trained to classify mental health problems. By analyzing mental-health-related data, as shown in Figure 3, the system helps healthcare monitoring systems automatically identify depression and anxiety such that patients will receive the social support they need.

RETRACTED

### 3.1. Data Collection

This section discusses the data collection procedure from two different sources. We collected our own data sets from Reddit and Twitter using common API wrappers, PRAW and Tweepy.  Figure 3 of task 1 shows the entire flow of data collection for the proposed framework. For Twitter, we selected appropriate words preceded by the hashtags symbol, which represents the main theme of content for specific topics. For the Reddit data, we focused on specific subreddits that were suitable for our targeted topics and then performed a search query on such topics. These platforms offer application programming interfaces (APIs) such as PRAW and Tweepy, which allow us to access the data.

### 3.2. Preprocessing

Data preprocessing is a method of cleaning and filtering noisy and vague data so that they can be easily used for feature extraction, as shown in Figure 4. In real world, people exchange information on social media in an informal way, with texts that contain hashtags, special characters, and needless words. We have to apply the concept of machine learning and data mining in order to extract some sense out of such text corpus before feeding them to any classification model. In addition, substituting jargon and emojis with the corresponding informative text using Emojipedia is the main area of our focus. It is well known that the Internet is becoming a communication medium where people frequently use colloquial speech and emojis to convey their opinions and thoughts. Extracting meaningful text from posts in social media helps understand the context and intensify the emotions associated with it. We applied different preprocessing methods to our collected text, which contain many jargons and informal words in a way it will help us identify depression and anxiety, as depicted in Figure 4.

#### 3.2.1. Tokenization

Tokenization is a method of splitting a sizable amount of text into smaller portions, commonly known as tokens. These tokens are utilized to discover some patterns and are taken as an input for the next common steps in the NLP pipeline, such as stemming and lemmatization, as shown in 1 of task 2. In general, a large text is composed of hash signs, punctuation, and characters that are not even texts. In our proposed system, this process is conducted using the TreebankWordTokenizer that is found in the natural language toolkit (NLTK) to purify the words called tokens. Tokenization is used to reduce nonalphanumeric characters and break down sentences into words. Finally, all the text in the entire given file is represented by a bag of words for further analysis.

RETRACTED

#### 3.2.2. Removing Stop Words

In this subsection, we discuss the removal of words that have no significant information on mental-health-related problems in general. The most frequent words considered irrelevant are pronouns, prepositions, symbols (e.g., dates, #), conjunctions, and articles (a, an, and the). In addition, universal resource locators (URLs) in any given text data should be filtered because they have no useful information in text processing. To remove stop words from a given sentence, we first split our text into words and then eliminate the word if it occurs in the list of stop words provided by the NLTK, as described above. Substituting jargon and emojis with their factual text using Emojipedia is an extremely critical step because they contain helpful information regarding mental health.

#### 3.2.3. Conversion to Lowercase

People usually present their opinions about how they feel using emojis. Some words may be written differently such as “b4,” that is, “before”; “):,” that is, “happy”; and “2moro,” that is, “tomorrow.” Each word in our scenario is converted into its original and generic form, followed by conversion into lowercase, which maintains consistency and avoids confusion during a text analysis.

#### 3.2.4. Part-of-Speech (POS) Tagging

The practice of categorizing words into their parts of speech and marking them accordingly is called part-of-speech tagging (POS). These labels can be nouns, verbs, adjectives, adverbs, determiners, and conjunctions, among others. The main reason behind this step is to discard any POS that has no contribution to the identification of depression and anxiety. In addition, POS tagging recognizes nouns and adjectives, which are considered invaluable indicators for sentiment analysis. We used the NLTK POS-tagger for our proposed system, as shown in Figure 4.

### 3.3. Text Representation

Word embedding is a technique used to represent words in a given text corpus with a real-valued vector that capture the meaning of the word such that the words that remain in a close neighborhood are anticipated to be identical in meaning. We implemented many word-embedding techniques to represent our collected text corpus (bag of words) into the equivalent vectors. Word vectors are much better ways to represent words than the older techniques, such as a one-hot encoded vector, where the index assigned to each word does not hold any semantic meaning. In addition, word vectors consume much less space than one-hot encoded vectors and also maintain a semantic representation of words. We have summarized many real-valued vector representation techniques, as shown in Figure 2, and most of them are implemented using Python 3.7. Figure 2 shows the word embedding techniques from the old context-free techniques such as word2vec and GloVe to bidirectional contextual representations such as BERT, ELMo, and OpenAI GPT [19, 20]. We propose the recent and smart method, BERT, to obtain the context of a given word in our collected text corpus.

RETRACTED

#### 3.3.1. Word2vec

The word2vec algorithm accepts a text corpus and generates an equivalent vector associated with the given input. The generated vector will have high dimensions, and each word included in the text will be given an associated vector in vector space. The vectors are placed in space such that words with similar contextual meaning will stay in closer proximity to one another. However, the word2vec algorithm is unable to represent a new word with a vector if it is not included in the training data set. As shown in Figure 5, the word2vec model has very famous architectures, that is, continuous bag-of-words and skip-gram, in which the training phase uses one hidden layer. However, the purpose of training each of them is different. CBOW is a model that finds a target word using neighboring context words, whereas the skip-gram model finds context words given a center word as an input. In our proposed system, the skip-gram model was trained to use its improved performance with consistent words. To find word representations that can infer adjacent words within a context *c* with high accuracy, the skip-gram model for a given series of words \{*w*_1_, *w*_2_, *w*_3_,… *w*_*n*_\} increases the objective of the average log probability over all *N* target words and their respective contexts.

(1) $$\begin{array}{c} \frac{1}{N}=\sum_{n=1}^{N}\sum_{-c⩽j⩽c_{j}\neq 0}\log\;P\left(w_{n+j}|w_{n}\right). \end{array}$$

The probability predicted for a given center word is highly dependent on the inner product of the vectors used to represent the input and output candidates \{*w*_*I*_ and {*w*_*O*_}, respectively, normalized to the requirements of a probability distribution over all words in the vocabulary of size *N* using the softmax function as follows:

(2) $$\begin{array}{c} P\left(w_{o}|w_{i}\right)=\frac{\exp\left(v_{w_{o}}^{T}v_{w_{I}}\right)}{\sum_{w=1}^{W}\exp\left(v_{w}^{T}v_{w_{I}}\right)}. \end{array}$$

However, the complexity of determining these probabilities and correlated gradients for all words becomes expensive as the size of the words increase. In most of the previous word embedding techniques depicted in Figure 2, the major drawback is extremely small context, and no global occurrence is used. For the entire data set collected from Reddit and Twitter, we passed each pair into the neural network and trained our model to represent the collected texts.

RETRACTED

#### 3.3.2. FastText Model

As the working principle of fastText, the morphological structure of a word contains key information about the meaning of the word. Such a structure was not exploited much by conventional word representation techniques such as word2vec, which trains a distinctive word representation for every single word in the list. This is more useful for morphologically rich languages where a given word may have a larger number of morphological forms, making it difficult to train good word embeddings. FastText tries to resolve this by considering each word as a collection of subwords. For simplification and language independence, subwords are considered as the character *n*-grams of the word. The vector for a word is simply considered as the sum of all vectors of its component char *n*-grams. Based on a comprehensive comparison of word2vec and fastText in our experiment, fastText performs considerably better on syntactical tasks as compared to the original word2vec, particularly when there is a smaller number of training data. word2vec marginally outperforms fastText on semantic tasks.

#### 3.3.3. BERT

BERT is a recent approach proposed by researchers using the Google AI language. BERT uses the transformer architecture, an attention mechanism that discovers contextual contacts between words [45]. The transformer contains two separate components: an encoder that reads the text input and a decoder that generates a prediction for the task. Because BERT's main target is to produce a language model, only the encoder mechanism is necessary. During training, BERT utilizes two schemes to capture the contextual meaning of words in both the right and left directions.

*(1) Masked Language Model (MLM)*. Before passing the input sequences into the BERT model, 15% of the words in each sequence were substituted with a [MASK] token. BERT then tries to infer the initial value of the masked words based on the context provided by the other words in the sequence. A prediction is conducted based on three main steps, as depicted in Figure 6:

- Applying a classification layer on top of the encoder output
- Multiplying the output vectors by the embedding matrix and transforming them into the vocabulary dimensions
- Computing probability distribution for all the words in the vocabulary using softmax

*(2) Next Sentence Prediction (NSP)*. During the training process, the BERT model takes two sentences and finds some correlation to predict if the second sentence is the follow-up (next sentence) of the first sentence in the original document. During the training phase, half of the input is a pairing in which the second sentence is the consequent sentence in the original document, and the other half of the input is a second sentence randomly selected from the text corpus.

RETRACTED

BERT uses an encoder from transformer architecture that is an encoder-decoder network based on self-attention on the encoder side and attention on the decoder side [45]. BERT is of two sizes: a base BERT (BERTBASE) and a large BERT (BERTLARGE). BERTBASE has 12 layers in the encoder stack, whereas BERTLARGE has 24 layers in the encoder stack. The BERT architectures (BASE and LARGE) also have larger feedforward networks (768 and 1,024 hidden units, respectively), and more attention heads (12 and 16, respectively) than the transformer architecture suggested in the original study [45]. It contains 512 hidden units and 8 attention heads. BERTBASE contains 110M parameters, whereas BERTLARGE has 340M parameters. This model takes the classification token (CLS) as the first input, followed by a sequence of words that are being forwarded to the next layer. Each layer applies a self-attention and passes the result to the next encoder through a feedforward neural network. We propose BERT-based word embedding and fine-tuning to our specific health-related problem task based on the hyperparameters described in Table 1.

### 3.4. Classifier Models

We implemented many recent state-of-the-art classifier models to create the last sentiment classification on our data set. In our experiment, we implemented an SVM, a logistic regression, a random forest, and AdaBoost. With deep learning techniques, words are represented as a dense vector, and a machine-learning-/deep-learning-based sentiment classification will be applied by passing dense vectors to the classification models. Recurrent neural networks (RNNs), which are the most common sequence modeling techniques, are capable of obtaining appropriate features from data and can be a leading choice for capturing the semantics of long texts. However, an RNN is somehow an inclined model because it allocates a high priority to recently appearing words in a sequence, which might lessen its efficiency when capturing the semantics of an entire document. As a result, LSTM was instituted to surmount the flaws in maintaining long-term dependencies in RNN models [36]. The LSTM model along with a convolutional neural network (CNN) for sentence classification provides accurate results and has been recently utilized in a variety of NLP tasks. CNN models use convolutional and maximum pooling layers to extract the most relevant features, whereas LSTM models maintain the relationship between words for a longer period using memory cells. Hence, they are better used for text classification [36, 47]. A bidirectional LSTM consisting of two such memories was developed to tackle sequence classification problems. As an example, it was applied in traffic event analysis along with OLDA using social networking data and achieved an extremely high accuracy [48]. Based on the results, We propose a bidirectional LSTM (Bi-LSTM), which uses two LSTM units, that works in both left and right directions to combine past and future context information from our collected social media data. Bi-LSTM also retains a long-term relationship between words along with duplicate context information, as depicted in Figure 7 [49].

RETRACTED

In each LSTM unit shown in Figure 7, there are hidden layers with the capability of keeping the previous information for a reasonably longer period. The LSTM architecture contains the main component called the memory cell {*c*_*t*_} that is being updated by using the input gate {*i*_*t*_} and forget gate {*f*_*t*_}, as shown in (4). The input gate {*i*_*t*_} is responsible for deciding which information should be stored in the memory cell. The forget gate {*f*_*t*_} is used to decide which information needs to be discarded from the memory cell. At each time step, {*c*_*t*_} for the forward LSTM can be updated using (4) as follows:

(3) $$\begin{array}{c} f_{t}=\sigma \left(\omega_{f}.\left(h_{t-1},x_{t}\right)+b_{f}\right),\\ C_{t-2}=\left(\text{tahnh}\left(w_{c}.h_{t-1},x_{t}\right)+b_{c}\right). \end{array}$$

(4) $$\begin{array}{c} C_{t}=f_{t}*c_{t-1}+i_{t}*C_{t-2}. \end{array}$$

(5) $$\begin{array}{c} o_{t}=\sigma \left(\omega_{o}.\left(h_{t-1},x_{t}\right)+b_{o}\right),\\ h_{t}=o_{t}*\;\tanh\left(C_{t}\right). \end{array}$$

In our proposed framework, we used a principal component analysis (PCA) before feeding the embedding vectors to the classifiers. PCA is a technique with the primary purpose of reducing the dimension of a data set consisting of many related variables, either heavily or lightly, while preserving the variation available in the data set. As it can be seen in Figure 8, we conducted intensive experimentation to exploit and compare the key advantages of each word embedding and classification technique, which have recently become extremely popular. Our research was conducted on Reddit and Twitter data, which are classifications of depression/anxiety-related posts (positive/negative) using deep-learning-based text analysis techniques.

We propose a two-way implementation approach, as it is depicted in Figure 8, the first of which is the implementation of state-of-the-art machine/deep learning techniques for depression/anxiety identification along with dimensionality reduction to maximize the accuracy. The second most important part is applying fine-tuning and model optimization (knowledge distillation) to build a lighter and smarter depression/anxiety detection model. Knowledge distillation here is building a compressed model by teaching it exactly what to do in a sequential manner using a larger pretrained BERT model [19]. Our proposed knowledge distillation-based sentiment analysis model is further described in Figure 9, which shows how pretrained weights from BERT are used are fine-tuned to our depression/anxiety detection downstream task to build a smarter and lighter model.

RETRACTED

The teacher-student architecture used throughout this research is a universal structure for knowledge transfer [41]. In other words, the quality of knowledge gain and extraction from teacher to student is also dependent on how the teacher-student network is designed. The guidance message from the larger model, which is known as “knowledge,” supports the smaller model to simulate the behavior of the larger complex model. In the sentiment analysis task, logits (e.g., the output of the last layer in a deep neural network) are used as a means to propagate knowledge from the teacher model, which is not clearly given by the training data sets. Given a vector of logits *z* as the output of the last fully connected layer of a deep model, such that {*z*_*i*_} is the logit for the *i*-th class, the probability {*p*_*i*_} that the input belongs to the *i*-th class can then be estimated using the softmax function as follows:

(6) $$\begin{array}{c} p_{i}=\frac{\exp\left(z_{i}\right)}{\sum_{j}\exp\left(z_{j}\right)}. \end{array}$$

Therefore, the predictions of the soft targets obtained by the teacher model include dark knowledge and can be utilized as a supervisor to migrate knowledge from the complex model to a simple one. In our proposed framework, we built a smaller student model from a pretrained (unsupervised) large BERT model using our collected data set (labeled data). Our proposed framework has the following key steps:

- Training the teacher model: the complex teacher network (BERT) is initially trained on a large generic data set (Wikipedia and BookCorpus). This phase demands high-performance computational environment such as high-performance GPUs.
- Establish correspondence: in constructing a student network (distilled BERT), there should be a connection between the immediate outputs the student and teacher models. This relationship can be done either by directly forwarding the output of a layer in the teacher network to the student network or doing data augmentation before passing it to the student network.
- Forward pass through the larger model: the data are forwarded through the teacher network to get all the immediate results and then apply data augmentation.
- Applying backpropagation: the result from the teacher network and the correlation is used to backpropagate the error in the student network.

RETRACTED

We used response-based knowledge, which usually refers to the result of the last output layer of the teacher model (last logits). Response-based knowledge distillation is known to be simple and effective for compressing large models and was commonly used in many NLP tasks recently. As described in Figure 9, the distillation loss of response-based knowledge can be formulated as follows:

(7) $$\begin{array}{c} L_{D}\left(p\left(z_{t}\right),p\left(z_{s}\right)\right)=L_{\text{KL}}\left(p\left(z_{s}\right),p\left(z_{t}\right)\right), \end{array}$$

where LKL is the Kullback–Leibler divergence loss. The Kullback-Leibler divergence score, or KL divergence score, quantifies the extent to which one probability distribution differs from another probability distribution. In our case, the KL divergence between two distributions *Q* (teacher model) and *P* (student model) is often stated using the following notation: KL(*P* – *Q*), where the – operator indicates a “divergence,” or the divergence of *P* from *Q*. KL divergence can be calculated as the negative sum of probability of each event in *P* multiplied by the log of the probability of the event in *Q* over the probability of the event in *P* as follows:

(8) $$\begin{array}{c} \text{KL}\left(P\|Q\right)=-\text{sum }x\text{ in }XP\left(x\right)*\;\log\left(\frac{Q\left(x\right)}{P\left(x\right)}\right). \end{array}$$

Based on this loss calculation, backpropagation takes place such that the student network can learn to replicate the behavior of the teacher network.

## 4. Experimental Results

The results of our proposed scheme are discussed in this section. The next remaining subsection describes the data set utilized to train and test the classification models. In Subsection 4.2, we introduce the methods used to effectively measure the performance of our classifier model, and the results will be explained in subsection 4.3. Finally, Subsection 4 describes the various experimental results achieved through our study.

### 4.1. Data Sets

We designed a data collection framework using Twitter and Reddit APIs (Tweepy and PRAW, respectively) to collect data on depression and anxiety, studied different text-based emotion detection techniques, and used the circumplex model of affect to use keywords belonging to different emotions, as shown in Figure 1 [50]. A common way to define a set of emotions can be using a list of words expressing each emotional trait. We used a keyword-based approach that is based on predetermining a set of terms to classify the text into emotion categories such as happy, angry, and sad, which were used to gather the most significant data on depression and anxiety from social media platforms. In our data set, we collected 100,000 tweets and 95,000 posts from Twitter and Reddit, respectively. One common problem in data preparation is using an imbalanced data set where data belonging to one class are significantly higher or lower in number than those belonging to other classes. As a result, the learning algorithm might choose to ignore those underrepresented classes. Therefore, we tried to balance the number of positive and negative classes (52% and 48%, respectively). We collected posts and comments from Reddit using two commonly applied subreddits called r/Depression and r/Anxiety and labeled them as positive, whereas the standard posts filtered by keywords based on the circumplex model shown in Figure 1 [30] are labeled as negative.

RETRACTED

Table 2 shows a summary of the data sets collected based on our proposed framework. We merged them together and prepared training and test data sets. We used word cloud to visualize frequent words in a text where the size of the words represents their frequency in the positive (depression-related posts) and negative (standard posts) directions collected using keywords related to happiness and excitement, as depicted in Figure 10.

### 4.2. Performance Matrices

To evaluate our model, we used the commonly used metrics, such as precision, recall, and accuracy. A confusion matrix is a matrix used for evaluating the classification performance, which is also called an error matrix because it shows the number of incorrect predictions versus the number of correct predictions in a tabulated manner. Based on the confusion matrix, we can compute the accuracy, precision, and recall as follows:

(9) $$\begin{array}{c} \text{precision}=\frac{\text{TP}}{\text{TP}+\text{FP}},\\ \text{recall}=\frac{\text{TP}}{\text{TP}+\text{FN}},\\ \text{accuracy}=\frac{\text{TP}+\text{TN}}{\text{TP}+N+\text{FP}+\text{FN}}. \end{array}$$

The most commonly used terminologies that are used in calculating the confusion matrix are as follows:

- P: an actual positive case, which is the depression-/anxiety-related class in our model
- N: an actual negative case, which is nondepression-/nonanxiety-related class in our model
- True positive (TP): a case in which the actual class of the data point (collected text data) is true (1), and the class predicted by our model is also true (1)
- True negative (TN): a case in which the actual class of the data point is false, and the predicted class is also false
- False positive (FP): a case in which the actual class of the data point is 0 (false), and the predicted class is 1 (true)
- False negative (FN): a case in which the actual class of the data point is true, and the predicted class is false

RETRACTED

### 4.3. Results

In the experiment we have conducted, we studied our model attributes along with numerical performance knowledge distillation-based model and state-of-the-art machine learning algorithms. We used two data sets, namely, depression- and anxiety-related text posts collected from social media specifically from Reddit and Twitter users.

#### 4.3.1. Our Proposed Approach versus State-of-the-Art Algorithms

In our experiment, the proposed Bi-LSTM and BERT-based knowledge distillation scheme were compared with RF, LG, SVM, CNN, AdaBoost, MLP, and LSTM algorithms for identifying depression-/anxiety-related sentiments using our own data as shown in Tables 3 and 4. We used an RF with 150 iterations, 100 estimators, and SVM with a training parameter ridge estimator and a radial basis function (kernel = rbf), respectively. In baseline algorithms, we use three famous word embedding techniques, such as TF-IDF, word2vec, and fastText that are applied on SVM, NB, RF, and AdaBoost models as shown in Table 3. Our main target here was to examine which feature extraction techniques best favor the performance for depression and anxiety detection based on our collected data. We applied 150 estimators and a learning rate of 0.8 as the hyperparameters in AdaBoost achieved an accuracy of 83%. In addition, we implemented SVM with a training parameter ridge estimator and a radial basis function (kernel = rbf), getting an accuracy of 84%. SVM works relatively well compared with AdaBoost because there is a clear margin of separation between labels given to each of the collected text corpora after preprocessing and vectorization. The performance in most of the classical machine learning algorithms in Table 3 is decreased while applying word2vec because the word2vec algorithm discards unseen words during the training phase.

Next, we have used a principal component analysis (PCA) to reduce the dimensionality of a data set consisting of many related variables, either heavily or lightly, while preserving the variation available in the textual data. We have used dimensionality reduction that involves reducing the number of input variables while we were generating vectors from the collected list of tokens. Fewer input variables can result in a simpler predictive model that have a better performance when making predictions on new data. As we have shown in the result section of our paper, for every vectorization method like BERT, GloVe, and word2vec, there were performance improvements because of PCA because of less number of parameters. As presented in Table 4, the accuracy of almost all classifiers increased when we apply principal component analysis as a dimensionality reduction, except for the case of random forest (RF), Naive Bayes (NB), and logistic regression (LR) when using the word2vec vector. It is because word2vec is unable to handle new words, and it influences these models to be inefficient in terms of accuracy.

RETRACTED

Table 5 presents the results obtained from the proposed Bi-LSTM, knowledge distillation, and five other classification algorithms. These classification models were used to predict mental-health-related problems using three types of text vectorization techniques such as word2vec, GloVe, and BERT, and the results of all baseline approaches were compared to assess the performance of the word vectorization models. Bi-LSTM and distilled BERT achieved higher classification accuracies of 96% and 98%, respectively. The main reason is that the student (distilled BERT) model mimics the teacher model that initially was trained on general text corpus such as Wikipedia and BookCorpus. Therefore, distilled BERT obtains a competitive or even a superior performance when fine-tuned to our depression- and anxiety-related data domain. The learning of this small model from the bigger pretrained model in our proposed framework is termed knowledge distillation. In addition, BERT outperforms word2vec and GloVe for both anxiety and depression prediction tasks because BERT is able to distinguish and capture two different semantic meanings by producing two different vectors for the same word in a given text corpus. We can see that Bi-LSTM with BERT can precisely infer depression and anxiety from a given large text corpus as shown in Table 5.

Figure 11 presents the comparison of accuracy and loss with respect to the training and testing phase of our proposed Bi-LSTM. We compared the training and test accuracy of the Bi-LSTM model with the BERT-based text representation as shown in Figure 11. We get training accuracy after applying the model on the training data, while test accuracy is the accuracy on the test data. We have run our experiment for 20 epochs both for model accuracy (a) and model loss (b) in Figure 11. We can see that they follow the same trend under different parameter settings (batch_size = 64, epochs = 20, verbose = 1, and validation_split = 0.2). This small difference between our training and test accuracy shows that we have a proper setting of the regularization of all parameters of the network and a well representative data batch. Finally, Table 1 presents the hyperparameters used in our repeated experiment. We have set optimal hyperparameters and optimizer algorithms used to train our models as shown in Table 1. The parameters used were batch size, epochs, optimizer, and number of hidden layers and Adam as an optimizer performed well in our experiment. We applied hyperparameter tuning by conducting a repeated experiment and applied these parameters to control the learning process. We have achieved the best accuracy under these parameter settings listed in Table 1.

RETRACTED

#### 4.3.2. Comparison with the Existing System

We compared our proposed system with the state-of-the-art systems, which were designed to analyze and predict mental-health-related problems from social media data, as presented in Table 6. Kim et al. utilized the word2vec model with XGBoost and a CNN for depression- and anxiety-related text classification and achieved an accuracy of 75.13% on depression-related data and 77.81% on anxiety-related data [28]. Mickael et al. presented depression detection techniques using combined features (LIWC + LDA + bigram), classifying them using SVM and MLP, and obtained accuracies of 90% and 91%, respectively [37]. Hatoon et al. applied linguistic inquiry and word count (LIWC) with a linear SVM to predict depression from Twitter data and obtained an accuracy of 82.50% [43]. Zogan et al. employed multimodalities + word embedding (word2vec) with a bidirectional gated recurrent unit-convolutional neural network (BiGRU-CNN) for depression detection from Twitter data and achieved an accuracy of 85% [26]. In 2019, Kumar et al. utilized a feature matrix with ensemble vote classification using RF, NB, and gradient boosting and obtained an accuracy of 85.09% [27]. The accuracy of our system is shown in the last row of Table 6. During this experiment, we adopted the concept of knowledge distillation using BERT and fine-tuned our task of depression and anxiety detection, obtaining an accuracy of 98% for anxiety-related data and 97% for depression-related data. In addition, we employed an attention mechanism to hold the long-term relationship among words using transformer architecture and applied Bi-LSTM to predict anxiety, obtaining an accuracy of 96%. The results obtained show that the proposed techniques might help in the development of smart and efficient systems for the detection of depression, anxiety, and other health-related problems from social media textual contents created by users.

## 5. Conclusion

In this study, we developed a strongly constructed framework for the detection of mental health problems using deep learning techniques such as BERT, Bi-LSTM, and a knowledge distillation based on social media content created by users. The proposed framework enhances the accuracy of smart healthcare systems to detect mental-health-related problems mainly depression and anxiety. This research work can be utilized to build a real-time system for early mental-health-related problem detection mainly based on user posts on Reddit and Twitter. We discussed various key features, including mental-health-related textual data collection from social networks using application programming interfaces and preprocessing module that focuses on the conversion of unstructured data into a meaningful form using various data filtering techniques. We also have employed a keyword and circumplex model-based text labeling technique on the collected text corpus to extract useful features related to mental health. Furthermore, our mental health problem detection framework applies the most recent text embedding technique based on deep learning that ensures capturing the semantic and contextual meaning of words included in user posts.

RETRACTED

The proposed BERT-based text representation model transforms collected words into vectors capturing the semantic meaning in the collected text corpus to improve the accuracy of the classification task using an attention mechanism. We also proposed response-based knowledge distillation, which is based on the neural response of the last output layer of the teacher model (last logits) in BERT for building a smaller and smarter model for depression/anxiety detection and classification. Moreover, we developed our own data collection module to prepare the data set from Twitter and Reddit by mining the most relevant textual data that can be used to build an intelligent model for smart healthcare systems. Finally, we conducted an intensive experiment, based upon which the proposed BERT-Bi-LSTM model improves the accuracy of text sentiment classification from user posts. The main reason the model outperforms other machine learning classification models is that it combines the strengths of both BERT and Bi-LSTM models to comprehend the syntactic and contextual information of each word. In addition, we implemented a response-based knowledge transfer using BERT, fine-tuned the task of depression/anxiety detection, and achieved extremely high accuracy. In future work, a multimodel depression detection system can be developed to utilize more diverse data such as text, image, and behavioral features to achieve effective results.

## Figures and Tables

**Figure 1:** Graphical representation of the circumplex model of affect with the horizontal axis representing the valence or pleasant dimension and the vertical axis representing the arousal or activation dimension.

RETRACTED

**Figure 2:** Different real-valued vector representation techniques for a predefined large-sized vocabulary from a corpus of text.

**Figure 3:** These layered schematic diagrams show an organized view of automatic detection of depression and anxiety from user posts. The data collection, preprocessing, and labeling layer deals with generating meaningful data from data sources such as Reddit and Twitter. The text vectorization and classification section deals with the technique of extracting meaningful insights from the labeled data using deep learning.

**Figure 4:** The basic natural language processing pipelines used while preparing data. We used these techniques to convert the collected text into small chunks so that they will be consumed by our machine learning model.

**Figure 5:** Word2vec embedding architecture with the skip-gram model. Both the input vector x and the output y are one-hot encoded word representations. The hidden layer is a word embedding of size *N*.

**Figure 6:** Masked language modeling used to train BERT, where a model uses the context words surrounding a mask token to try to predict what the masked word should be.

**Figure 7:** Bi-LSTM process used to capture sequential features.

**Figure 8:** Our proposed general framework for text representation, dimensionality reduction, and depression/anxiety detection based on fine-tuning and knowledge distillation techniques along with the common feature-based classification.

**Figure 9:** Detailed architecture of applying knowledge distillation from pretrained BERT to build a smaller task-specific model on health-related problem identification.

**Figure 10:** Depression-related posts (left) versus standard posts (right) using a word cloud.

**Figure 11:** Comparison of training and test accuracy (a) versus training and test loss (b) for proposed Bi-LSTM model. The parameters we have used for the experiment were batch_size = 64, epochs = 20, verbose = 1, and validation_split = 0.2.

**Table 1:** Hyperparameters used in the deep learning techniques in our experimental environment.

Hyperparameters	Deep learning model				
	CNN	LSTM	Bi-LSTM	BERT fine-tuning	Proposed KD-based classification
Batch size	64	64	64	4	4
Epochs	20	20	20	3	3
Optimizer	Adam	Adam	Adam	Adam	Adam
Number of hidden layers	128	128	128	768	768

**Table 2:** Description of the data sets collected from Reddit and Twitter.

Data sources	Mental health problems	Collected posts	Description
Reddit	Depression	75,000	Discussions and posts related to depression
	Anxiety	80,000	Discussions and posts related to anxiety
Twitter	Depression	25,000	Contents and posts related to depression
	Anxiety	15,000	Content and posts related to anxiety

RETRACTED

**Table 3:** Performances of classical machine learning algorithms with our collected data (A, accuracy; P, precision; and *R*, recall in %).

Classification models																				
Embedding techniques	*NB*			SVM			RF			MLP			LR			DT			AdaBoost		
	A	P	R	A	P	R	A	P	R	A	P	R	A	P	R	A	P	R	A	P	R
Tf-IDF	82	83	81	84	84	84	83	82	82	83	82	83	83	83	83	83	82	82	83	83	82
Word2vec	67	67	67	73	73	74	73	73	73	82	82	82	70	70	70	68	69	68	74	74	74
FastText	67	69	65	84	84	83	78	79	78	86	86	86	80	79	78	77	76	77	83	83	82

**Table 4:** Performances of classical machine learning algorithms with our collected data after applying a PCA.

Classification models																				
Embedding techniques	NB			SVM			RF			MLP			LR			DT			AdaBoost		
	A	P	R	A	P	R	A	P	R	A	P	R	A	P	R	A	P	R	A	P	R
Tf-IDF	82	83	81	84	84	84	83	82	83	83	82	83	83	83	83	83	82	82	83	83	82
Word2vec	60	57	59	75	74	74	71	72	68	80	80	80	69	68	70	71	71	68	75	75	75
FastText	69	67	64	85	85	85	80	80	80	86	86	86	80	79	78	77	76	77	82	82	82

Values written in bold are the best recorded performance (accuracy) of our algorithm.

**Table 5:** Deep-learning-based text representation and classifier models applied to our generated data set including our proposed scheme.

Embedding methods	Classification models						
	MLP	SVM	LSTM	Bi-LSTM	1-D CNN	BERT_fine-tuning	Proposed KD distilled_BERT
	Accuracy	Accuracy	Accuracy	Accuracy	Accuracy	Accuracy	Accuracy
Data sets used-depression-related data (depressed vs. normal)							
GloVe	82%	78%	87%	88%	84.50%	—	—
BERT	90.32	90.35	89%	91.34	87%	90%	**97%**

Data sets used-anxiety-related data (anxiety related vs. normal)							
Word2vec	90%	88%	94.20%	**96%**	94.30%	—	—
BERT	91%	85%	95.80%	**96%**	94.30%	**96%**	**98%**

**Table 6:** Detailed comparison of existing methods for the detection of depression-/anxiety-related data on social media.

Author (year)	Data source	Word embedding model	Classifiers	Overall accuracy
Jina Kim (2020)	Reddit	Word2vec (form gensim)	XGBoost and CNN	75.13% (depression) 77.81% (anxiety)
Michael (2019)	Reddit	LIWC + LDA + bigram (combined feature)	SVM and CNN	90% and 91%, respectively
Hatoon (2020)	Twitter	LIWC Sentiment analysis	Linear SVM	82.50%
Tadesse (2020a)	Reddit	Word2vec	LSTM-CNN	93.80%
Akshi Kumar (2019)	Twitter	Feature matrix	Ensemble vote, classification (RF, NB, and B)	85.09%
Hamad (2020)	Twitter	Multimodalities + word embedding (word2vec)	BiGRU-CNN	85%
Our proposed approach	Reddit and Twitter	Word2vec, fastText, and BERT	LSTM, Bi-LSTM, and BERT + knowledge distillation	94%, 96%, and 98%, respectively

RETRACTED

## Data Availability

The data sets used for mental health prediction are available from the corresponding author upon request.
